The article "Forecasting the Severity of COVID-19 Pandemic Amidst the Emerging SARS-CoV-2 Variants: Adoption of ARIMA Model" was published in 2022. Journal: Comput Math Methods Med.

# Forecasting the Severity of COVID-19 Pandemic Amidst the Emerging SARS-CoV-2 Variants: Adoption of ARIMA Model

**DOI:** 10.1155/2022/3163854

**Published:** 2022-01-13

**Authors:** Cai Li, Agyemang Kwasi Sampene, Fredrick Oteng Agyeman, Brenya Robert, Abraham Lincoln Ayisi

**Affiliations:** ^1^School of Management, Jiangsu University, Zhenjiang 212013, China; ^2^College of Economics and Management, Nanjing Agricultural University, Nanjing 210095, China; ^3^School of Finance and Economics Zhenjiang, Jiangsu 212013, China

## Abstract

Currently, the global report of COVID-19 cases is around 110 million, and more than 2.43 million related death cases as of February 18, 2021. Viruses continuously change through mutation; hence, different virus of SARS-CoV-2 has been reported globally. The United Kingdom (UK), South Africa, Brazil, and Nigeria are the countries from which these emerged variants have been notified and now spreading globally. Therefore, these countries have been selected as a research sample for the present study. The datasets analyzed in this study spanned from March 1, 2020, to January 31, 2021, and were obtained from the World Health Organization website. The study used the Autoregressive Integrated Moving Average (ARIMA) model to forecast coronavirus incidence in the UK, South Africa, Brazil, and Nigeria. ARIMA models with minimum Akaike Information Criterion Correction (AICc) and statistically significant parameters were chosen as the best models in this research. Accordingly, for the new confirmed cases, ARIMA (3,1,14), ARIMA (0,1,11), ARIMA (1,0,10), and ARIMA (1,1,14) models were chosen for the UK, South Africa, Brazil, and Nigeria, respectively. Also, the model specification for the confirmed death cases was ARIMA (3,0,4), ARIMA (0,1,4), ARIMA (1,0,7), and ARIMA (Brown); models were selected for the UK, South Africa, Brazil, and Nigeria, respectively. The results of the ARIMA model forecasting showed that if the required measures are not taken by the respective governments and health practitioners in the days to come, the magnitude of the coronavirus pandemic is expected to increase in the study's selected countries.

## 1. Introduction

Recently, there have been different reports globally concerning the variant of severe acute respiratory syndrome coronavirus 2 (SARS-CoV-2) family that spreads even quicker than the coronavirus disease 2019 (COVID-19) [1]. In Wuhan, China, a new virus (COVID-19) was detected in December 2019. The COVID-19 has spread throughout China and the rest of the world [2, 3]. Coronaviruses are highly contagious and rapidly transferred from person to person. The disease, which is now a global pandemic, has spread swiftly around the world, causing severe public health issues as well as an economic crisis. When unpredictable infectious diseases arise, causing an outbreak leads to an epidemic and eventually results in a pandemic [4]. Researchers attempt to use modelling techniques to explain the observable trends and predict specific patterns in the future so that health practitioners can organize health care programs, and their responses can be planned to mitigate such situations [4, 5]. Wangari et al. [6] noted that epidemiological models are becoming increasingly useful for understanding the complex processes regulating infectious disease transmission.

Phan [7] reported that one of the characteristics of COVID-19 is its highly pathogenic nature and possibly a zoonotic agent that quickly spreads among people, which makes it very dangerous for the world and needs proper measures put in place to curb or control the spread by each country. Scientists are putting in measures by actively conducting empirical studies to make relevant decisions concerning COVID-19 that may end the pandemic. Anjorin [8] reported that the risk to global public health, including the extreme acute threat in 2002, is an outbreak of respiratory syndrome (SARS) that caused 800 deaths with approximately 8000 reported cases. Emerging infectious diseases continue to threaten humanity and cause many deaths, which reduce the world population drastically. According to estimates, the H1N1 pandemic of 2009 killed 18500 people; 800 people out of 2500 cases in 2012 died from the Middle East Respiratory Syndrome (MERS) [8, 9]. Ebola outbreak killed 11310 people out of 28616 cases in 2014, and the latest coronavirus disease (COVID-19) pandemic has killed more than 2.43 million people out of 110 million reported cases [8, 9]. This research focuses on four countries (United Kingdom, South Africa, Brazil, and Nigeria). The reason for selecting these countries was because, according to a report by the Center for Disease Control and Prevention (CDC), these countries recorded the first recorded cases of the SARS-CoV-2 new variant [10]. The ending section of the year 2020 saw many countries around the globe recording different forms of SARS-CoV-2. According to a report released by the Centers for Disease Control and Prevention (CDC) in December 2020, several SARS-CoV-2 variants are circulating worldwide [10].

In the United Kingdom (UK), a new variant of COVID-19 (B.1.1.7) was detected in early 2021. Volz et al. [11] noted that the SARS-CoV-2 variant B.1.1.7 spread across the United Kingdom early this year. The Visual and Data Journalism Team [12] observed that there is a recent spike in coronavirus cases, and this increase is driven by the new variant (B.1.1.7). This lineage B.1.1.7 possesses a large amount of no-synonymous substitution of immunological significance. The World Health Organization report indicated that variant B.1.1.7 had spread globally to more than 50 countries [13, 14]. Rendana and Idris [14] reported that there had been reported new cases of about 50000 of the variant B.1.1.7 in the UK since it started speeding among the populace in the early part of this year.

Volz et al. [11] observed that the mortality rate of COVID-19 would rise due to the new variant. Similarly, Horby et al. [15] found that the COVID-19 variant B.1.1.7 is related to a higher risk of death than different variants. More quickly and rapidly than other varieties, this version spreads faster than COVID-19. Among 60-year-olds in the UK, the coronavirus death rate was around 10 per 10,000. Nevertheless, the UK currently records about 13 or 14 deaths in the same population with the new strain. Different symptoms from those associated with the original COVID-19 virus are often dominated by the more recent variant [16].

Brazil (BRA) publicly announced the emergence of the SARS-CoV-2 variant (P1) or “gamma” in January this year [17]. The SARS-CoV-2 variant P1 has evolved, and health experts in Brazil suggested that the variant might contribute to the rise in the number reported in Manaus. The gamma lineage has a mutation that helps it control a person's antibodies from previous infections, which indicates that there is a high possibility that it can easily reinfect people who had already had coronavirus [17]. Silva et al. [18] reported that the new COVID-19 variant P1 might increase the risk of respiratory infections, increase the death rate, and even lead to the collapse of health care in Brazil. Similarly, Page and Hambly [17] opined that, compared to the original SARS-CoV-2 virus, the gamma coronavirus variant has several mutations, including the N501Y mutation, which is also present in the alpha or B.1.1.7 variant and the beta or B.1.351 variant. This mutation makes it easier for the virus's spike proteins to bind to human cells, potentially making it more infectious. Madhi et al. [19] also indicated that the UK strain B.1.1.7 has been associated with an increase of 53% transmissibility rate.

The variant P1 adds to the worries since it seems to have hit a similar constellation of mutations and has appeared in a position with a high immunity level. In a case of a group in the Amazon region, Sabino et al. [20] found that 42% of the specimens sequenced from late December were correlated with the P1 variant. The area has, however, observed an increase in cases since mid-December. The advent of this variant poses questions about a possible rise in the transmissibility or tendency of individuals to reinfect SARS-CoV-2 [10].

South Africa (SA) health authorities reported a new variant of SARS-CoV-2 called B.1.351 (N501Y.V2). South Africa has also reported a new COVID-19 strain that appears to have mutated more than the UK's variant. B.1.351 was first discovered in early October 2020 and shared specific mutations with B.1.1.7. This new strain may be responsible for driving the country's current resurgence of the disease, although it is too early to confirm it. As the number of total confirmed cases exceeds one million, South African authorities have imposed stricter restrictions. According to health officials and scientists heading the country's virus strategy, this version is dominant among newly reported infections in South Africa. It tends to be more infectious than the original virus [10].

A recent report by Mwenda et al. [21] indicated that variant B.1.351 was first found in the Eastern Cape Province of South Africa. The detection of the South Africa B.1.351 coincided with the rise in coronavirus new cases in Zambia, which is close to South Africa. The B.1.351 variant may be linked to higher viral loads, and it contains another spike protein mutation that may prevent antibody binding, reduce vaccine efficacy, or blunt naturally developed immunity [21]. The B.1.351 variant is a cause for concern because it has increased disease transmission and decreased vaccine efficacy. There may be some form of improved immune pressure escape and onward transmission in B.1.351, resulting in a strength and conditioning advantage, but the evidence for this is still lacking [22].

The Nigeria Center for Disease Control (NCDC) confirmed that varying variants of SARS-CoV-2 are recognized to be percolating in Nigeria (NIG) as of February 14, 2021, and are rapidly evolving. The variation of SARS-CoV-2 strains suggests multiple virus introductions into Nigeria from various parts of the world, and it adds to evidence of community transmission in different Nigerian states [23]. A new version of SARS-CoV2 that has been recorded in Nigeria is the most recent discovery. From the other mutations, it is of a different lineage. The first B.1.525 case in Nigeria was discovered in a sample taken from a patient in Lagos State. As a result, B.1.525 is a new strain but not yet a variant of concern, and more research is underway [23]. In mid-December, B.1.525 was first discovered by genome sequence in Nigeria, but cases quickly followed in the United Kingdom, France, and other countries. B.1.525 represented over 20% of Nigerian genomes sequenced after only two months. Haseltine [24] reported that there have been over 200 reported cases of Nigeria variant B.1.525 around the globe.

Mathematical models have been identified as critical techniques that can help provide a framework for our understanding of infectious diseases [4]. Statistical methods can be used to model and forecast COVID-19 transmission. The obtained forecasts should be used to execute controlling techniques and make necessary decisions to mitigate the impact of COVID-19 [25]. Among the several univariate time series methodologies, Autoregressive Integrated Moving Average (ARIMA) and exponential smoothing techniques are commonly used for modeling. Aljandali [26] indicated in a recent study that statistical and forecasting models such as ARIMA and Seasonal Autoregressive Integrated Moving Average (SARIMA) for time series predictions for infectious disease patterns have been widely used and give accurate results. One of the most pressing issues in dealing with pandemics like COVID-19 is early detection and a short-term estimate of the pandemic's eventual magnitude and peak time. Early prediction using mathematical and statistical models combined with existing data will successfully assist governments and public health experts in implementing suitable preventative and control initiatives [27].

Using the ARIMA model, Ceylan [28] predicted the pattern of coronavirus emergence in the most affected European nations, specifically France, Spain, and Italy. The study results offered insight into the epidemic's patterns and explained these regions' epidemiological levels. Predicting coronavirus incidence trends in Italy, Spain, and France could also aid other countries in preparing for the outbreak by assisting them in developing policies and precautions. To forecast the COVID-19 epidemiological data of reported daily cases, Perone [29] used the ARIMA model to analyze the COVID-19 epidemiological data of confirmed daily cases in Italy. The ARIMA model was used by Lman et al. [30] to forecast COVID-19 incidence in some African countries. The study's results indicated that the virus's spread would intensify in the coming days.

Furthermore, Ding et al. [31] studied the forecasts for Italy's new confirmed and death cases. Their research proposed a time series analysis for the predictions based on the ARIMA model and discovered that the COVID-19 spread surge forecast could be realized with a preprocessed cumulative newly diagnosed scenario based on the ARIMA and FUZZY time series methodologies. Verma et al. [32] developed some models for predicting COVID-19 infections, mortality, and recovery in India and Maharashtra. The estimated values for Maharashtra and India as a whole were in exceptional alignment with actual values in all six COVID-19 scenarios.

Moreover, Yonar [33] forecasted the numbers of coronavirus pandemic cases in Turkey and particular G8 countries using ARIMA and other prediction models. This study indicated that certainly, more precise assessments could be made in future studies with more data. However, as this study provides data on the number of cases that may be increased in the absence of action in the current situation, it may direct countries to take the appropriate steps and intervene earlier.

The various literature reviewed indicated that the ARIMA model is more suitable for predicting pandemics like the coronavirus. The ARIMA model is one of several predictive methods that allow scientists to estimate and forecast the frequency and pattern of an event like COVID-19. The ARIMA and SARIMA models for disease prevalence have been employed by an outsized variety of researchers reducing outbreaks of various diseases [2, 31, 34–37]. COVID-19 pandemic has affected the world economy in different phases, leading to partial lockdown and total lockdown for some countries and the closure of factories worldwide; physicians, politicians, business people, operational directors, scientists, and civilians alike are all in disarray. Effective prediction of COVID-19 case trends is crucial for preparing the proper health care delivery system for affected individuals and the country in terms of pandemic management and resource planning.

The contribution of this study is that we innovatively used the ARIMA model to estimate whether SARS-CoV-2 will increase amidst the new COVID-19 variant reported in these countries. The study is aimed at helping monitor the pattern of the COVID-19 and the new variant of SARS-CoV-2 in the selected countries. The ARIMA model was chosen for forecasting in this study because it theoretically justifies the forecasting and optimizes the prediction performance of the COVID-19 variant. Likewise, the forecast also provides a formidable data platform to help the respective government or health professionals of the countries selected to make prudent decisions concerning the prevalence or spread of the pandemic.

This paper is organized as follows.  Section 2 describes the materials and methods used in this study.  Section 3 reports on the results of the article. The discussion of this study is embedded in Section 4. Concluding and recommendations are outlined in Section 5.

## 2. Materials and Methods

### 2.1. Description of Data

The research study period extends from March 1, 2020, to January 31, 2021 (337 days). This present study depends on daily cases and death cases of COVID-19 data gathered from (https://covid19.who.int). We fitted the model with the new cases and death cases due to the continued increase in the global recorded new case of COVID-19, which better can predict the trend. Moreover, the authors selected the new reported and death cases in this research to anticipate the future prevalence of COVID-19 in the specified countries. Through the lens of the new cases and death, it provides the raw data on the ground to enable policymakers to draw counter programs and policies to seal the source of infection emergence. Furthermore, several researchers, for instance [2, 38–41], used the daily new cases and death cases in the forecasting of COVID-19 cases around the globe.

The case definition by the World Health Organization for SARS-CoV-2 variant infection is as follows:

- First, a patient must meet the criteria for a diagnosis and be a contact related to a suspected or confirmed case
- Second, there is a suspected case with symptoms indicative of COVID-19 illness on chest imaging
- Third, a person has recently developed anosmia (loss of smell) or ageusia (loss of taste) with no other known causes
- Finally, an adult with respiratory distress before death who was a contact of a possible or confirmed case or associated with a COVID-19 cluster died for no apparent reason [42]

The case definition for new COVID-19 cases refers to a viral test as the only way to designate a COVID-19 case as “confirmed.” If one tests positive, it is referred to as a “confirmed COVID-19 case.” This indicates that the person is afflicted with COVID-19 and is hence infectious. If a viral test comes out negative, the person is not currently infected with COVID-19 [43]. For monitoring purposes, a COVID-19 death is defined as a death in a probable or confirmed COVID-19 case caused by a clinically compatible illness, unless a clear alternative cause of death cannot be linked to COVID-19 disease (e.g., trauma). There should be no time for total recuperation [43].

#### 2.1.1. United Kingdom

The current population of the UK hovers around 68 million as of November 2021 [44]. The first case of coronavirus in the United Kingdom was recorded on January 31, 2020. Currently, the UK has recorded over 9 million COVID-19 cases as of November 2021, with more than 140,000 death cases [45].  Figure 1 indicates a graphical representation of new confirmed cases and death cases between March 1, 2020, and January 31, 2021.

#### 2.1.2. South Africa

South Africa is a historically and culturally prosperous nation positioned at the African continent's southern tip, bordering the Indian and South Atlantic Oceans. With a population of 56.5 million citizens, the region is a one-of-a-kind example of economic development, with several new advances that are more relevant than one might expect [46]. South Africa confirmed the first case of COVID-19 on March 5, 2020. As of November 2020, South Africa has recorded over 2 million COVID-19 instances, with more than 80,000 deaths recorded.  Figure 2 indicates a graphical representation of new confirmed cases and death cases for South Africa between March 31, 2020, and January 1, 2021.

#### 2.1.3. Brazil

Brazil's first record of COVID-19 was on January 3, 2020. Brazil is one of the countries hardest hit by the COVID-19 pandemic, with over 21 million confirmed cases and over 600000 confirmed deaths by November 2021 [47]. The beginning of 2021 was marked by the second wave of COVID-19, which differed from the first wave, with simultaneous explosive surges of COVID-19 cases across different regions of the country, adding enormous pressure to a health system already under strain after a year of the pandemic [48].  Figure 3 indicates a graphical representation of new confirmed cases and death cases for Brazil between March 31, 2020, and January 1, 2021.

#### 2.1.4. Nigeria

On February 27, 2020, the first case was confirmed in Nigeria. More than 200000 reported cases and over 2000 deaths as of November 2021 [38]. COVID-19 testing rates in Nigeria have been significantly lower than in other African countries with comparable population sizes. This has been linked to delays in a testing kit and reagent supplies during border closures [38].  Figure 4 indicates a graphical representation of new confirmed cases and death cases for Brazil between March 31, 2020, and January 1, 2021.

### 2.2. ARIMA Model

The Autoregressive Integrated Moving Average (ARIMA) models, developed by Box and Jenkins in the 1970s, are time series models commonly used today for predictions and making a relevant decision with the forecasted values [49]. ARIMA is a time sequence model that is based on a given time series data. The three terms that make up an ARIMA model are **p**, **d**, and **q**, where **p** stands for the order of the autoregressive (AR) expression, **q** for the order of the moving average term (MA), and **d** for the amount of difference required to correct the time arrangement. The difference's base number is the **d** estimate, which is expected to correct the disparity.

The ARIMA model involves a complicated process, but it can be summarized in these four steps:

- Identification of the ARIMA structure (**p**, **d**, **q**)
- Estimation of the coefficient of the formulation
- Diagnostic test or fitting test of the estimated residuals
- Forecasting the future outcomes based on the historical data

The autoregressive (AR) model involves regressing the variable of interest of *Y*_*t*_ on its lagged values *Y*_*t*−1_, *Y*_*t*−2_, ⋯*Y*_*t*−*p*_. The moving average (MA) process includes regressing the time series *Y*_*t*_ on the current residuals *ε*_*t*_ and its lagged residual *ε*_*t*−1_, *ε*_*t*−2_, *ε*_*t*−3_, ⋯, *ε*_*t*−*q*_. The integrated (*I*) denotes the difference between the actual time series data and its lagged values. The differencing can be done once or twice [9]. The ARMA (**p**, **d**, **q**) model is typically expressed mathematically as follows:

(1) $$\begin{array}{c} Y_{t}=\alpha +\varphi_{1}\;Y_{t-1}+\varphi_{2}\;Y_{t-2}+\cdots +\varphi_{p}Y_{t-p}+\varepsilon_{t}-\theta_{1}\varepsilon_{t-1}-\varepsilon_{t-2}-\cdots -\theta_{1}\varepsilon_{t-q}, \end{array}$$

where *φ* and *θ* are the AR and MA parameters and *α* is the constant term in the model. *Y*_*t*_ represents the confirmed and death cases at a day, and *t* denotes the date of the first case of COVID-19 detected in a given country. *ε*_*t*_ are the values of the residual at time *t* such that *ε*_*t*_ ~ *N*(0, *σ*^2^). The time series plot of the daily COVID-19 confirmed cases and death cases for all the selected countries is presented in Figures 1–4, respectively.

### 2.3. Akaike Information Criterion (AIC) and Akaike Information Criterion Correction (AICc)

The main issue with ARIMA modeling is choosing the best ARIMA model. Based on the model selection criteria, the best ARIMA models can be found. Model selection criteria typically used in ARIMA models include Akaike Information Criterion (AIC) and Akaike Information Criterion Correction (AICc). AIC provides a method for prediction accuracy. AIC estimates the corresponding volume of information lost by a given model: the less relevant data a model loses, the higher the model's quality. In forecasting the volume of data lost by a model, AICc considers the trade-off between the model's goodness of fit and its simplicity. Sen and Shitan [50] reported that model selection aims to discover a good predictor that describes a system. The Akaike Information Criterion (AIC) and AICc are standard model selection approach in the ARIMA model [50].

(2) $$\begin{array}{c} \text{AIC}=-2\;\ln\;\left(\text{L}\right)+2K,\\ \text{AICc}=\text{AIC}+\frac{2\left(k+1\right)\left(K+2\right)}{n-k-2}, \end{array}$$

where *L* is the model's likelihood and *K* denotes the total number of estimated parameters. A good model is one with the lowest AIC among all other models.

### 2.4. Criteria for the Comparison of Goodness-of-Fit

The AR and MA expressions have been combined in an ARIMA model, which means the time series has been differentiated at least once to make it stationary. To determine the accuracy of our model, we performed three tests: root mean square error (RMSE), mean absolute error (MAE), and mean absolute percentage error (MAPE).

(3) $$\begin{array}{c} \text{MAE}=\frac{1}{n}\overset{n}{\underset{i=1}{\sum }}{\left|Y_{I}-\overset{\wedge }{Y_{i}}\right|}^{\prime },\\ \text{MAPE}=\frac{100}{n}\times \overset{n}{\underset{i=1}{\sum }}{\left|Y_{I}-\overset{\wedge }{Y_{i}}\right|}^{\prime },\\ \text{RMSE}=\sqrt{\overset{n}{\underset{i=1}{\sum }}\frac{\left(\hat{Y_{i}}-Y_{i}\right)2}{n}}, \end{array}$$

in which between *Y*_*I*_ the actual values and $\hat{Y_{i}}$ are the predicted values of the ARIMA model at time *t*.

## 3. Results

The ARIMA model used for the research was first examined with the Augment Dickey-Fuller Test to check the data's stationarity. The Autocorrelation Function (ACF) and Partial Autocorrelation Function (PACF) plots test the ARIMA model parameters. PACF estimations are used to depict the model during the evaluation process since they have different characteristics. The ACF for AR (**p**) falls off at the order of *p*, but the PACF remains constant; for MA (**p**, **q**), neither the ACF nor the PACF tails off. The ARIMA model predicts values with upper and lower bounds, and an estimated value 1-*α* point confidence interval exists between the upper and lower limits. Any realization that falls within the gap will be accepted, according to the provided confidence.

The Ljung-Box (Q18) was used to assess the model fitness and determine how well it can make better predictions. The ARIMA model was used to forecast confirmed and death cases for the selected countries over the next 27 days to see if the current COVID-19 variant would increase confirmed new and death cases. MAPE values and root mean square error (RMSE) were evaluated to check the forecast's accuracy and validity.

### 3.1. Descriptive Statistics for the Selected Countries

The descriptive statistics from the study indicate that an average of 4314, 16645, 27314, and 389 people have contacted the COVID-19 virus in South Africa, U.K, Brazil, and Nigeria, respectively. Also, an average of 131, 306, 666, and 5 people have succumbed to the COVID-19 pandemic in South Africa, U. K, Brazil, and Nigeria, respectively. The data's skewness values for both confirmed new and daily confirmed death cases were more than one except for Brazil. This means that the daily reported cases and death cases are skewed to the right, as indicated in Table 1.

### 3.2. Unit Root Test (Augmented Dickey-Fuller Test)

The Augmented Dickey-Fuller (ADF) Test was used to verify that the time series was stationary (daily confirmed new cases and confirmed COVID-19 death cases). The test results are shown in Table 2. At the level difference of the ADF test, daily new cases and death cases of the data were not stationary. However, data for both confirmed new cases and daily confirmed death cases for each of the countries chosen became stable at the first level difference. As a result, the series is ready to be modeled with the Box-Jenken ARIMA mathematical model.

### 3.3. Autocorrelation Function (ACF) and Partial Autocorrelation Function (PACF)

The data were tested for stationarity and seasonality using the Autocorrelation Function (ACF) and Partial Autocorrelation Function (PACF) graphs. According to He and Tao [51], the PACF graph depicts the degree of correlation between a variable and a lag of that variable, where the correlation does not justify the low order lags. A diagnostic check of the fitted model residuals is required, which involves graphical analysis and statistical testing. The fitted model, histogram, ACF, and PACF were plotted to perform a visual investigation of residuals as indicated in Figures 5 and 6. Correlogram or ACF plots demonstrate that there is no autocorrelation of the residual error. We used the following diagnostic testing tools, ACF and PACF, to check the noise terms independence of the ARIMA model. A sequence plot of the residuals, the ACF, and the PACF sample showing the residuals from these ARIMA models follow the white noise method. Therefore, the estimated ARIMA model can capture the dependent structure of the new confirmed new cases and time series of death cases very well.

We then analyzed the parameters for the selected ARIMA models to check the coefficient of the MA and AR components of the model, standard error (s.e.), Akaike Information Criterion (AIC), Akaike Information Criterion Correction (AICc), and the *P* value. The study used an ARIMA model with a minimum AICc and significant parameters. Accordingly, for the new confirmed cases, ARIMA (3,1,14), ARIMA (0,1,11), ARIMA (1,0,10), and ARIMA (1,1,14) models were chosen for the UK, South Africa, Brazil, and Nigeria, respectively, with a minimum AICc of 4805.208, 6682.536, 7626.332, and 5024.805. The *P* values were also statistically significant for the model. Also, the model specification for the confirmed death cases, ARIMA (3,0,4), ARIMA (0,1,4), ARIMA (1,0,7), and ARIMA (Brown) models were selected for the UK, South Africa, Brazil, and Nigeria, respectively, with AICc of 2826.250, 4384.203, 5034.412, and 2081.057. The *P* values of the AR and MA were statistically relevant with parameters of 0.05, meaning that the variables are significantly different from zero at the 95 percent confidence interval. The parameters also suggest that the selected model is the best for forecasting, as indicated in Table 3.

We then analyzed the parameters for the selected ARIMA models to check the coefficient of the Moving Average (ma) and autoregression component of the model, standard error (s.e.), Akaike Information Criterion, Akaike Information Criterion Correction (AICc), and the *P* value. The study used an ARIMA model with a minimum Akaike Knowledge Criterion Correction (AICc) and significant parameters. For the new cases of COVID-19 time series data, the best models selected for all the countries were UK ARIMA (3,1,14), South Africa ARIMA (0,1,11), Brazil ARIMA (1,0,10), and Nigeria ARIMA (1,1,14), respectively, with a minimum Akaike Information Criterion Correction (AICc) of 4805.208, 6682.536, 7626.332, and 5024.805. The *P* values were also statistically significant for the model. With regard to the death cases, the ARIMA model specification selected UK ARIMA (3,0,4), South Africa ARIMA (0,1,4), Brazil ARIMA (1,0,7), and Nigeria ARIMA (Brown), respectively, with minimum Akaike Information Criterion Correction (AICc) of 2826.250, 4384.203, 5034.412, and 2081.057. The *P* values of the AR and MA were statistically relevant with parameters of 0.05, meaning that the words are significantly different from zero at the 95% confidence interval stage. The parameters also suggest that the selected model is the best for forecasting.

Table 4 displays the goodness of fit criteria values of the Box-Jenkins statistics for each selected nation for confirmed new cases and daily confirmed death cases. Generally, the models have high *R*^2^ values for confirmed new cases and daily confirmed death cases. The *R*^2^ values for confirmed new cases for the selected countries were 0.971, 0.952, 0.712, and 0.877 for South Africa, the UK, Brazil, and Nigeria. The *R*^2^ values for confirmed death cases for the selected countries were 0.134, 0.205, 0.705, and 0.804 for South Africa, Brazil, and Nigeria. The *P* value of the Box-Jenkins statistics for the model is very significant and shows that the ARIMA model selected is the best fit for forecasting.

The mean absolute percentage error (MAPE), which transforms absolute errors into a percentage of actual numbers, is a better measure of forecast performance. The MAPE was lowest in the UK, followed by South Africa, Brazil, and Nigeria, suggesting that the forecast follows the linear pattern and confirms the estimates' accuracy. For the confirmed new cases, MAPEs for the UK, South Africa, Brazil, and Nigeria were 25.390, 28.867, 32.958, and 36.186. Also, for the predicted death cases, the mean absolute percentage errors (MAPE) were 60.955, 46.651, 30.343, and 80.946 for the UK, South Africa, Brazil, and Nigeria, respectively, as presented in Table 4.

### 3.4. Forecasting

Following the estimation of the ARIMA model for each country, we forecasted new cases and death cases for the selected countries over the next 27 days, thus from March 1, 2021, to March 27, 2021. The Ljung-Box test indicated that the expected values closely matched the actual values. The modified and forecast values are shown in Tables 5 and 6. Countries like the UK, South Africa, and Brazil had an unprecedented increase in possible COVID-19 incidents.  Figure 7 indicates a graphical representation of the forecasted values for confirmed new cases and death cases for the selected countries.

## 4. Discussion

We noticed from the forecasting that 95% confidence interval confirmed cases for all the countries selected for the studies might be between 21633 and 49637, 5264 and 16684, 1003 and 1936, and 42736 and 80043 for the UK, South Africa, Nigeria, and Brazil, respectively. For the death cases, the forecasted values revealed that the cases might be between 819 and 1439, 243 and 705, 16 and 26, and 930 and 1782 for the UK, South Africa, Nigeria, and Brazil, respectively. This study supports the recent findings of Horby et al. [15], who reported that the COVID-19 variant B1.1.7 is related to a higher risk of death than other variants.

The results indicate that the spread of the new variant of SARS-CoV-2 will increase the number of new cases in the UK. Also, concerning the death cases, analysis from the paper shows that if health officials and the government do not implement proper measures, the new variant will cause an increase in the death toll in the UK. A recent report by Betsy KIein [52] indicated that the UK variant B.1.1.7 is more contagious than the original strain (COVID-19), and it is also possibly more dangerous and associated with a higher risk of death. In Brazil, the study showed that there would be an increase in the number of confirmed new cases, as indicated in Table 5. Death cases in Brazil resulting from the coronavirus are expected to rise based on the analysis of this study. This result supports Taylor [53] in which this report estimated that almost 400000 Brazilians have died from COVID-19, indicating a 13% of the world's total COVID-19 deaths, which is even more than the country's entire AIDS epidemic.

Also, in South Africa, forecasting from the study revealed that new coronavirus cases would be appreciated in the days ahead. Death cases resulting from COVID-19 will be a bit lower than those in countries like the UK and Brazil. Researchers have indicated that the South Africa variant (B.1351) may be approximately 50% more contagious based on the faster rate of the virus's structure that appears to make it simpler to infect human cells [54].

Interestingly, analysis from the study portrayed that in Nigeria, the prevalence of coronavirus daily cases may be slower than in the UK, Brazil, and South Africa. The death cases resulting from coronavirus are expected to reduce based on the results from this study. Ogundokun et al. [55] indicated that the Nigerian government made the right decision in enforcing the traveling restriction. This is because the results from their analysis revealed that traveling history and contact increase the chance of people being infected with coronavirus by 85% or 88%. The implication for the lower death rate may be because of stricter measures employed by the government in Nigeria. To the best of our knowledge, this is the first study to implement an ARIMA model to predict the incidence of COVID-19 in these countries since the new variant SARS-CoV-2 started spreading. The researchers perceived an increase in the prevalence of COVID-19 in the days ahead. If not handled by the government and health professionals, the death cases will escalate, and many people may continue to die from the virus.

## 5. Conclusion and Recommendation

COVID-19 has caused a lot of havoc and damage to humanity on the globe. Recently, several researchers have been attempting to examine the effects of COVID-19 on the economies of various countries and continents and forecast the virus's spread, existence, and other issues related to this pandemic. In this paper, the researchers looked at time series data for daily cases confirmed and daily deaths confirmed of the novel coronavirus and SARS-CoV-2 variants recently spread across the world. In the UK, South Africa, Brazil, and Nigeria, the ARIMA model examined daily and death cases. Daily confirmed cases and daily confirmed death cases for these countries from March 1, 2020, to January 31, 2021, were selected for the prediction using the ARIMA model.

The ARIMA model was chosen for this paper's study because of its widespread acceptance in the research field and the ease with which various stakeholders may act on these predictions. The study results show that the death cases in Nigeria are declining, which indicates that the government and experts have managed the situation well to achieve this feat. The other countries advised that firm measures need to be set up to curtail the virus from spreading. The researchers conclude that with the emergence of the novel COVID-19 variant spreading globally, if the necessary steps are not implemented to curb the prevalence rate, it is expected that there will be an increase in the new cases and death in the coming days of the selected countries.

Some practical recommendations suggested from the study to control the pandemic include the following: (i) the general public should be adequately informed about the coronavirus pandemic and its consequences for public health; (ii) expansion of the various health facilities in these countries has effective and efficient treatment and management of COVID-19 cases in the various hospitals in the selected countries; (iii) this paper would support the public health professionals in the respective countries to make prudent decisions concerning the prevalence of the pandemic; and (iv) proper measures should be put in place for testing and tracing of COVID-19 cases.

Finally, the researchers suggest that citizens in these countries must follow all the COVID-19 protocols (physical distancing, face-covering with nose masks, hand hygiene, coughing or sneezing hygiene, etc.). Various governments in these selected countries should put plans to educate the citizens on the need to take the coronavirus vaccination to help reduce the prevalence of COVID-19 in these countries and the rest of the world. Adhering to these measures will go a long way to help save humanity and the globe for a better living. Future work will be focused on the consequences of coronavirus mutations at the population levels to help policymakers implement measures to curb the prevalence of COVID-19 in the world.

## Figures and Tables

**Figure 1:** The new confirmed cases and death cases between March 1, 2020, and January 31, 2021, for the United Kingdom.

**Figure 2:** A graphical representation of new confirmed cases and death cases between March 1, 2020, and January 31, 2021, for South Africa.

**Figure 3:** A graphical representation of new confirmed cases and death cases for Brazil, between March 1, 2020, and January 31, 2021.

**Figure 4:** A graphical representation of new confirmed cases and death cases for Nigeria between March 1, 2020, and January 31, 2021.

**Figure 5:** The estimated ACF and PACF graphs to predict the epidemiological trend of new COVID-19 cases prevalence for (a) United Kingdom, (b) Brazil, (c) Nigeria, and (d) South Africa.

**Figure 6:** The estimated ACF and PACF graphs to predict the epidemiological trend of COVID-19 death case prevalence for (a) United Kingdom, (b) Brazil, (c) South Africa, and (d) Nigeria.

**Figure 7:** Graphical representation of future values forecasts for (a) the United Kingdom, (b) Brazil, (c) Nigeria, and (d) South Africa.

**Table 1:** Descriptive statistics on daily confirmed new cases and daily confirmed new death cases for South Africa, United Kingdom, Brazil, and Nigeria.

Countries	Cases	Minimum statistic	Maximum statistic	Mean statistic	Std deviation	Skewness statistic	Kurtosis statistic
South Africa	New cases	0.000000	21980.00	4313.831	4872.204	1.426217	4.368313
	Death cases	0.000000	844.0000	131.0504	160.9850	2.121297	7.824333

United Kingdom	New cases	0.000000	68192.00	16444.83	14810.52	1.654796	5.198443
	Death cases	0.000000	1826.000	306.3628	380.4005	1.523536	4.937794

Brazil	New cases	0.000000	87843.00	27313.74	19764.55	0.326550	2.190322
	Death cases	0.000000	1703.000	666.1068	422.4255	0.043674	1.961550

Nigeria	New cases	0.00000	2464.000	389.4392	416.4691	1.871882	6.774957
	Death cases	0.000000	0.000006	4.706231	5.281345	1.545259	5.766038

**Table 2:** ADF Test at level and difference 1 for the selected time series data.

Country	Model type	Transformation	Dickey-Fuller Test	Lag order	*P*
United Kingdom	New cases	Level Difference1	-1.899189 -17.32530	4 4	0.3326 ≤0.001^∗^
	Death cases	Level Difference1	-1.471263 -6.183466	4 4	0.8376 ≤0.001^∗^

South Africa	New cases	Level Difference1	-2.485075 -3.920069	4 4	0.8376 ≤0.001^∗^
	Death cases	Level Difference1	-1.471263 -6.183466	4 4	0.8376 ≤0.001^∗^

Brazil	New cases	Level Difference1	1.523484 -25.18564	4 4	0.8448 ≤0.001^∗^
	Death cases	Level Difference1	-1.448902 -26.38912	4 4	0.8448 ≤0.001^∗^

Nigeria	New cases	Level Difference1	-0.336076 -14.43101	4 4	0.9894 ≤0.001^∗^
	Death cases	Level Difference1	-2.616215 -14.10239	4 4	0.2734 ≤0.001^∗^

**Table 3:** Selected ARIMA model specification.

Country	Model type	Coefficient	Estimate	s.e.	AIC	AIC (AICc)	Likelihood	*P*
United Kingdom	New cases ARIMA (3,1,14)	ar3 ma1 ma7 ma14	-0.138 0.266 -0.270 -0.189	0.055 0.051 0.053 0.053	4805.151	4805.208	-2400.576	0.012 ≤0.001 ≤0.001 ≤0.001
	Death cases ARIMA (3,0,4)	ar1 ar2 ar3 ma1 ma2 ma3 ma4	0.546 -0.537 0.981 -0.242 -0.362 0.368 0.370	0.024 0.029 0.024 0.061 0.062 0.060 0.060	2826.193	2826.250	-1411.097	≤0.001 ≤0.001 ≤0.001 ≤0.001 ≤0.001 ≤0.001 ≤0.001

South Africa	New cases ARIMA (0,1,11)	ma2 ma4 ma6 ma7 ma11	0.113 0.114 -0.204 -0.400 0.218	0.050 0.054 0.051 0.051 0.056	6682.500	6682.536	-3339.250	0.024 0.034 ≤0.001 ≤0.001 ≤0.001
	Death cases ARIMA (0,1,4)	ma1 ma4	0.488 0.239	0.046 0.047	4384.203	4384.203	-2190.083	≤0.001 ≤0.001

Brazil	New cases ARIMA (1,0,10)	ar1 ma1 ma7 ma10	0.996 0.792 -0.322 0.264	0.006 0.038 0.032 0.031	7626.332	7626.332	-3811.166	≤0.001 ≤0.001 ≤0.001 ≤0.001
	Death cases ARIMA (1,0,7)	ar1 ma1 ma3 ma4 ma6 ma7	0.994 0.691 0.166 0.195 -0.244 -0.167	0.006 0.042 0.054 0.054 0.055 0.056	5034.376	5034.412	-2515.18	≤0.001 ≤0.001 0.002 ≤0.001 ≤0.001 0.003

Nigeria	New cases ARIMA (1,1,14)	ar1 ma2 ma7 ma14	-0.729 0.399 -0.355 -0.208	0.048 0.058 0.052 0.059	5024.805	5024.840	-2510.402	≤0.001 ≤0.001 ≤0.001 ≤0.001
	Death cases ARIMA (Brown)	Level and trend	0.064	0.009	2081.021	2081.057	-1038.511	≤0.001

**Table 4:** The goodness-of-fit criteria of the ARIMA model (Box-Jenkins).

Country	Model statistics								Ljung-Box (Q18)		
	Model type	Stationary *R*^2^	*R* ^2^	RMSE	MAPE	MAE	MaxAPE	Normalized BIC	Statistics	DF	*P*
United Kingdom	New cases ARIMA (3,1,14)	0.134	0.971	2505.822	25.390	1194.057	1912.005	15.750	29.110	12	0.004
	Death cases ARIMA (3,0,4)	0.860	0.860	141.294	60.955	81.110	1350.324	10.014	413.202	11	≤0.001

South Africa	New cases ARIMA (0,1,11)	0.337	0.952	1074.397	28.867	607.300	1244.993	14.044	108.426	13	≤0.001
	Death cases ARIMA (0,1,4)	0.205	0.784	74.721	46.651	39.896	550.064	8.661	211.774	16	≤0.001

Brazil	New cases ARIMA (1,0,10)	0.712	0.712	10715.299	32.958	7390.316	252.310	18.627	218.426	14	≤0.001
	Death cases ARIMA (1,0,7)	0.705	0.705	233.234	30.343	163.986	185.523	11.007	186.154	12	≤0.001

Nigeria	New cases ARIMA (1,1,14)	0.412	0.877	146.608	36.186	90.432	480.824	10.044	19.850	14	0.135
	Death cases ARIMA (Brown)	0.804	0.443	3.938	80.946	2.566	1267.098	2.758	19.427	17	0.305

**Table 5:** Prediction based on the ARIMA model of new cases for the selected countries at 95% confidence interval level for the next 27.

Model type	United Kingdom ARIMA (3,1,7)			South Africa ARIMA (0,1,11)			Nigeria ARIMA (1,1,14)			Brazil ARIMA (1,0,10)		
Date	Forecast	LCL	UCL	Forecast	LCL	UCL	Forecast	LCL	UCL	Forecast	LCL	UCL
3/1/2021	19843	14428	25873	4582	-26	6023	1045	745	1345	46699	25059	63820
3/2/2021	21464	14969	28790	4616	-595	6545	1417	1096	1739	54244	32178	68340
3/3/2021	22096	14999	30165	4642	-1058	7026	1171	837	1504	55110	32630	76310
3/4/2021	22587	14884	31422	4661	-1567	7167	1149	798	1500	49839	26956	77590
3/5/2021	21526	13556	30788	4680	-1572	7766	1397	1033	1760	47791	24514	72722
3/6/2021	20264	12113	29877	4728	-1552	8676	873	495	1252	41100	17439	71068
3/7/2021	19653	10869	30235	4738	-2307	9494	1198	770	1626	40411	14291	64761
3/8/2021	19475	10058	31025	4772	-2500	10687	967	519	1414	40008	11659	66530
3/9/2021	20193	9960	32893	4797	-3122	11319	1230	747	1713	45728	15327	68357
3/10/2021	20550	9684	34190	4817	-3957	11637	992	488	1496	45557	14691	76130
3/11/2021	20982	9487	35558	4836	-4341	12020	1080	547	1612	45386	14066	76422
3/12/2021	20576	8755	35787	4883	-4707	12387	1057	503	1611	45215	13452	76705
2/13/2021	20531	8293	36469	4893	-5059	12738	965	387	1543	45046	12847	76979
3/14/2021	20559	7722	37556	4927	-5397	13076	1032	415	1649	44877	12252	77244
3/15/2021	20702	7268	38755	4953	-5723	13402	983	340	1625	44708	11667	77501
3/16/2021	20796	6822	39846	4972	-6038	13717	1019	344	1693	44540	11090	77750
3/17/2021	20879	6426	40846	4991	-6343	14023	992	292	1693	44373	10522	77991
3/18/2021	20946	6047	41795	5039	-6640	14319	1011	283	1740	44207	9962	78225
3/19/2021	21020	5696	42730	5049	-6929	14608	998	245	1751	44041	9410	78451
3/20/2021	21096	5366	43652	5083	-7209	14889	1008	229	1786	43875	8866	78671
3/21/2021	21174	5056	44556	5108	-7483	15163	1000	198	1802	43711	8329	78885
3/22/2021	21250	4764	45441	5128	-7751	15430	1006	180	1831	43547	7800	79092
3/23/2021	21327	4489	46309	5147	-8012	15692	1002	154	1850	43383	7277	79294
3/24/2021	21403	4228	47161	5194	-8268	15948	1005	134	1875	43220	6762	79489
3/25/2021	21480	3982	47999	5204	-8519	16198	1003	111	1894	43058	6253	79679
3/26/2021	21556	3749	48824	5238	-8764	16444	1004	91	1917	42897	5750	79864
3/27/2021	21633	3528	49637	5264	-9005	16684	1003	70	1936	42736	5254	80043

**Table 6:** Prediction based on the ARIMA model of death cases for the selected countries at 95% confidence interval level for the next 27.

Model type	United Kingdom ARIMA (3,0,4)			South Africa ARIMA (0,1,4)			Nigeria ARIMA (Brown)			Brazil ARIMA (1,0,7)		
Date	Forecast	LCL	UCL	Forecast	LCL	UCL	Forecast	LCL	UCL	Forecast	LCL	UCL
3/1/2021	1226	389	1596	219	166	463	12	4	20	769	307	1230
3/2/2021	1130	856	1507	217	179	513	12	4	20	883	400	1365
3/3/2021	770	753	1159	217	208	576	12	4	20	1016	514	1518
3/4/2021	1017	381	1428	219	227	625	12	4	20	1104	599	1610
3/5/2021	1252	607	1672	219	223	629	12	4	21	1142	635	1648
3/6/2021	894	831	1321	220	219	633	13	5	21	1104	597	1611
3/7/2021	815	466	1258	223	215	637	13	5	21	1050	536	1565
3/8/2021	1194	372	1652	226	211	641	13	5	21	1044	505	1583
3/9/2021	1092	736	1556	224	207	645	13	5	21	1038	476	1599
3/10/2021	756	628	1229	224	204	649	13	5	22	1031	448	1615
3/11/2021	999	282	1488	226	200	652	13	5	22	1025	421	1630
3/12/2021	1212	509	1710	226	196	656	14	5	22	1019	394	1644
3/13/2021	868	714	1371	228	193	659	14	5	22	1013	369	1657
3/14/2021	804	364	1320	231	189	663	14	5	23	1007	345	1669
3/15/2021	1163	287	1691	234	186	666	14	5	23	1001	321	1680
3/16/2021	1055	634	1589	231	182	670	14	5	23	995	298	1691
3/17/2021	741	522	1283	232	179	673	14	5	23	988	275	1702
3/18/2021	980	200	1535	233	176	677	14	5	24	982	253	1711
3/19/2021	1173	425	1735	233	172	680	15	5	24	977	232	1721
3/20/2021	843	612	1409	235	169	683	15	5	24	971	211	1730
3/21/2021	792	276	1370	238	166	686	15	5	25	965	191	1738
3/22/2021	1132	215	1719	241	163	689	15	5	25	959	171	1746
3/23/2021	1020	545	1612	239	160	693	15	5	25	953	152	1754
3/24/2021	728	429	1326	239	156	696	15	5	25	947	133	1761
3/25/2021	961	129	1571	241	153	699	15	5	26	942	115	1768
3/26/2021	1136	351	1752	241	150	702	16	5	26	936	97	1775
3/27/2021	819	520	1439	243	147	705	16	5	26	930	79	1782

## Data Availability

We used the World Health Organization Covid-19 data which is freely available: https://covid19.who.int database.
